# Genetic Polymorphisms in miR-137 and Its Target Genes, TCF4 and CACNA1C, Contribute to the Risk of Bipolar Disorder: A Preliminary Case-Control Study and Bioinformatics Analysis

**DOI:** 10.1155/2022/1886658

**Published:** 2022-09-22

**Authors:** Mohammad Ali Mokhtari, Saman Sargazi, Ramin Saravani, Milad Heidari Nia, Shekoufeh Mirinejad, Kinga Hadzsiev, Judit Bene, Mansoor Shakiba

**Affiliations:** ^1^Department of Clinical Biochemistry, School of Medicine, Zahedan University of Medical Sciences, Zahedan 98167-43463, Iran; ^2^Cellular and Molecular Research Center, Research Institute of Cellular and Molecular Sciences in Infectious Diseases, Zahedan University of Medical Sciences, Zahedan 98167-43463, Iran; ^3^Department of Medical Genetics, Clinical Center, Medical School, University of Pécs, Pécs H-7624, Hungary; ^4^Department of Psychiatry, Zahedan University of Medical Sciences, Zahedan 98167-43463, Iran

## Abstract

Accumulating evidence has suggested that miR-137 and its target genes, CACNA1C, and TCF4, are amongst the most robustly implicated genes in psychiatric disorders. This preliminary study is aimed at investigating the effects of genetic variations in miR-137 (rs1625579A/C), TCF4 (rs1261084C/T), and CACNA1C (rs10774053A/G and rs10466907G/T) on BD susceptibility. We recruited 252 BD patients and 213 healthy subjects as the control group. Genotyping was performed using PCR-RFLP and ARMS-PCR methods. Enhanced risk of BD was found under the codominant homozygous, dominant, and allelic models of TCF4 rs1261084C/T, codominant homozygous and allelic models of CACNA1C rs10466907G/T polymorphisms, as well as codominant homozygous, dominant, recessive, and allelic models of the CACNA1C rs10774053A/G. Moreover, both TT/AG/GT/AA and TT/GG/GT/AC genotype combinations strongly increased the risk of BD in the participants. The bioinformatics analyses revealed that rs1261084C/T and rs10466907G/T created and disrupted binding sites of some miRNAs in the 3′-untranslated region of TCF4 and CACNA1C genes. In contrast, the rs10774053A/G created a new binding site for a major splicing factor and might have an effective role in the function of the CACNA1C protein. We have found that all the studied SNPs are positively associated with BD susceptibility. Replicated studies on different ethnicities are required to confirm these findings.

## 1. Introduction

Bipolar disorder (BD), also known as manic depression, is a severe mood disorder characterized by recurrent episodes of mania, depression, and abnormally elevated mood, which affect thought, perception, emotion, and social behavior [1]. Challenges like suicidal behavior, family devastation, psychological problems, and hospitalization have made BD a significant public health concern [2]. Most studies have reported 12-month estimates of approximately 1% for BD in European countries [3]. The Global Burden of Disease Study 2013 (GBD 2013) estimated 32.7 million cases of BD in 1990. However, by 2013, that number had increased to 48.8 million, a 49.1 percent rise in BD prevalence due to population growth and aging [4]. Results from the Global Burden of Disease Study 2017 showed that the disability-adjusted life years (DALYs) surged by 54.4 percent in BD patients, from 6.02 million in 1990 to 9.29 million in 2017.

With age-standardized incidence rate (ASIR) and age-standardized DALYs rate (ASDR) being lowest in East Asia and highest in tropical Latin America [5]. An epidemiological survey of psychiatric disorders in 2005 reported that the prevalence rate of bipolar mood disorder (BMD) was 0.96% in Iranians. Also, the prevalence of mood disorders was found to be 4.29%, with major depressive disorder (2.98%) having the highest incidence among mood disorders [6]. Still, for many parts of the world, including Iran, there has been limited or no prevalence data available [7].

Generally, BD is categorized into two subtypes: type I of BD (BDI) BDI and type II of BD (BDII) BDII. Patients with BDI experience at least one episode of mania or depression. In addition, they can also experience hypomanic and mixed episodes. Patients with BDII, on the other hand, mostly present hypomania and major depressive episodes. [8]. Growing evidence implies that some genetics and environmental factors influence the risk of BD, making it a multifactorial disease [9]. The precise etiology of BD has remained unclear; however, twins and adopted are exposed to a higher incidence for BD development [10]. More importantly, family history is among the most substantial risk factors affecting susceptibility to BD and implies crucial genetic and phenotypic complexity [11].

Meta-analysis of BD genome-wide association studies (GWASs) has discovered that many single nucleotide polymorphisms (SNPs) are associated with an enhanced risk of this mental disorder [12–14]. However, until 2013, these variations accounted for little inherited risk in Europeans [15]. Following the first GWAS of BD in 2007, several loci, including NCAN, ANK3, and CACNA1C, were found to be associated with BD risk, and these findings were later confirmed by some population-based genetic association studies [11, 13, 16].

Increasing evidence has shown that noncoding RNAs (ncRNAs), like microRNAs (miRNAs), are likely to contribute to the etiology of psychiatric disorders, such as BD [17]. In this respect, differential expression of some miRNAs has been detected in prefrontal regions of patients with schizophrenia (SCZ) or BD as compared to healthy individuals [18, 19]. Reports have already established that SCZ and BD share some overlapping genetic factors and abnormalities in the structure and function of the brain [20, 21]. Moreover, BD tends to resemble SCZ from the prospect of several genetic variations with low minor allele frequencies (MAFs) [22].

miRNAs are a broad subgroup of small ncRNAs that regulate gene expression through posttranscriptional mechanisms [23]. The nervous system has the broadest miRNA expression profile among all human tissues, with the most well-known miRNAs expressed in the neurons [24]. Some evidence suggests that miRNAs regulate the human brain's function and development [25]. Different studies have reported dysregulation of miRNAs in brain samples of BD patients [26–28].

miR-137, as an abundant microRNA in the brain, is crucial for controlling synaptic development, neuronal proliferation and differentiation, and the fates of embryonic neural stem cells (NSCs). As a result of its dysregulation, the neurological system's network that controls gene expression is altered, leading to mental illnesses [29]. miR-137 is highly expressed in synapses in the cortex and hippocampus of adult humans [30, 31]. It has been established that the upregulation of miR-137 in the dentate gyrus of patients with SCZ or BD [31]. Hence, normal expression of miR-137 is required for modulating neuronal proliferation and differentiation [32]. Some of the putative miR-137 target genes, such as CUB and Sushi multiple domains 1 (CSMD1), C10orf26 [now WBP1L], transcription factor 4 (TCF4), Zinc Finger Protein 804A (ZNF804A), and *α*1c-subunit of the L-type calcium channel (CACNA1C), have also shown significant correlation with BD. These genes have been confirmed as miR-137 targets by *in vitro* methods [33]. In addition, gene sets of possible miR-137 targets, including target sets implicated in axonal guidance signaling, Ephrin receptor signaling, long-term potentiation, PKA signaling, and Sertoli cell junction signaling, were enriched with variations associated with the risk of psychiatric diseases, such as SCZ [34]. Recent evidence has suggested the extensive polygenic overlap between risk phenotypes and BD and SCZ. In this connection, identifying specific loci associating with this shared risk helps understand physiologically feasible pathways that may explain risk-taking in patients with severe psychiatric disorders [35]. Because of this shared genetic backgrounds, miR-137 may also serve as a new player in BD. Therefore, the role of this miRNA and its downstream genes in regulating networks involved in neural development and brain function of BD patients is worth investigating.

Mainly, CACNA1C has been introduced by GWASs as a risk factor for the onset and development of BD [17, 36]. The CACNA1C gene encodes the *α* subunit of the voltage-dependent L-type calcium channel Cav1.2 protein [37]. Many recent reports have been published on the association between CACNA1C SNPs and behavior, neurogenesis, and risk of psychiatric disorders such as SCZ, BD, and depression. Their findings suggested a common genetic profile among them [17, 38, 39]. Therefore, CACNA1C genetic variations have ranked among the most conclusive genetic findings in such disorders [40]. On the other hand, the TCF4 gene encodes a transcription factor involved in developing a subset of neuronal progenitors. It has been shown that TCF4 overexpression resulted in SCZ-associated behaviors in transgenic mice [41, 42].

We have previously shown that various SNPs located in candidate genes could interact with adverse life events and greatly influence the risk of developing psychiatric disorders [43–47], including BD [48]. In the current study, for the first time, we aimed to evaluate the association between SNPs located within miR-137 (rs1625579A/C) and its target genes TCF4 (rs1261084C/T) and CACNA1C (rs10774053A/G and rs10466907G/T) and the risk of BD in an Iranian population.

## 2. Materials and Methods

### 2.1. Participants and Sample Collection

This case-control study was conducted on 252 subjects with BD referred to Baharan psychiatry hospital, Zahedan, Iran. The control group comprised 213 unrelated healthy subjects recruited by general advertisement through local community groups. These subjects have no family history of neuropsychiatric disorders or drug abuse. A clinical interview was used to exclude potential controls with BD based on criteria provided by the Diagnostic and Statistical Manual of Mental Disorders, Fifth Edition (DSM-V). Diagnosis of BD patients was made according to the diagnostic criteria provided in DSM-V as per the structured clinical interview [49, 50]. Two board-certified psychiatrists carefully examined these cases. Patients diagnosed with major depressive disorder, cyclothymic disorder, SCZ spectrum disorder, panic disorder, anxiety disorder, borderline personality disorder, substance use disorder, attention-deficit/hyperactivity disorder (ADHD), and related neuropsychiatric disorder were excluded. All subjects were adjusted regarding age, gender, and body mass index (BMI).

### 2.2. DNA Extraction and Genotyping

About 5 mL of the peripheral blood sample was drawn from all subjects in both case and control groups and collected into ethylenediaminetetraacetic acid- (EDTA-) contained tubes. DNA extraction was carried out using the salting-out method [51]. The restriction fragment length polymorphism-polymerase chain reaction (RFLP-PCR) technique [52] was used for genotyping both rs1261084C/T and rs10774053A/G SNPs. In addition, an amplification-refractory mutation system polymerase chain reaction (ARMS-PCR) [53] was applied to detect rs10466907G/T and rs1625579A/C variants. Information regarding the primer's sequences [designed via GeneRunner program (available from http://www.generunner.net/)] and the size of products are shown in Table 1.

For detecting all studied SNPs, the PCR reaction was performed with the predenaturation step at 95°C for 5 min, 35 cycles of denaturation at 95°C for 30 s, annealing at an appropriate temperature (based on Table 1) for 30 s, an extension at 72°C for 30 s, followed by a final extension step at 72°C for 5 min. The reaction tubes contained 10 *μ*L of Taq DNA polymerase 2× Master Mix (Pars Tous Biotech Company, Iran), 0.7 *μ*L of each primer (10 pm/*μ*L) (GenFanavaran Biotech company, Iran), 0.6 *μ*L of genomic DNA, and 8 *μ*L of deionized water, reaching a final volume of 20 *μ*L. For detection of rs1261084C/T, 10 *μ*L of the PCR product was incubated with 1 *μ*L of the FokI restriction enzyme (10 U/*μ*L, Fermentas, Germany) and 2 *μ*L of a 10× CutsMart buffer (in a total 20 *μ*L reaction) overnight at 37°C. As for rs10774053A/G, 10 *μ*L of PCR product of was digested by 1 *μ*L of MspI (10 U/*μ*L, Fermentas, Germany) restriction enzyme and incubated with 9 *μ*L of 10× Buffer Tango at 37°C for 16 hours, with the same reaction volume. The final fragments were separated through electrophoresis in 2% agarose gels stained with DNA Green Viewer (Pars Tous, Company, Iran) and visualized using an ultraviolet light system (Figure 1). For quality control, approximately 25% of the samples were randomly genotyped, and genotyping accuracy was 100%.

### 2.3. Statistical Analysis

Data were analyzed using the SPSS package for windows, V22.0 (IBM Corporation, Armonk, NY, USA). To calculate the sample size, we first performed a pilot study by collecting the blood samples of a small population (100 subjects, including 50 BD patients and 50 healthy subjects) and genotyping the four SNPs. Next, the allelic frequencies of the SNPs in both groups were determined using the Chi-square test. The calculated frequencies were then analyzed using an online sample size calculator server (available at: https://clincalc.com/stats/SampleSize.aspx) [54]. The server uses the following formula for calculating sample size.

(1) $$\begin{array}{c} n=\frac{{\left(z_{1-\alpha /2}+z_{1-\beta }\right)}^{2}\left(P_{1}\left(1-P_{1}\right)+P_{2}\left(1-P_{2}\right)\right)}{{\left(P_{1}-P_{2}\;\right)}^{2}}, \end{array}$$

where,

*P*_1_ represents the frequency of the wild or mutant allele in control, *P*_2_ is the frequency of the wild or mutant allele in case, *Z* is the critical *Z* value for a given *α* or *β*, *α* indicates the probability of type I error (usually 0.05), and *β* is considered the probability of type II error (usually 0.2).

With study power set to 80%, the sample size was calculated for the tested SNPs in studied groups via the calculator. The threshold of sample size was then adjusted to a total of 465 subjects. Deviations from HWE in cases and controls were examined using the Chi-square (*χ*^2^). Quantitative data were reported as the mean and standard deviation and expressed as numbers and/or percentages. Statistical differences between data sets were analyzed using multivariate logistic regression, the independent *t*-test, or the Mann–Whitney test, where appropriate. The *χ*^2^ test was also used to calculate differences between the genotypic and allelic frequencies of the subjects in the studied population. The odds ratios (ORs) and the 95% confidence intervals (CIs) were similarly measured. A *p* value <0.05 was considered statistically significant.

### 2.4. Computational Analyses

Computational analyses were performed to investigate the impact of studied SNPs on the different aspects, including secondary structure of transcripts, miRNA binding sites, splicing sites, and protein function. For this purpose, the mirSNP database, as a collection of human SNPs in predicted miRNA target sites, was used to detect the effect of SNPs on the miRNA binding sites [55]. The SpliceAid2 database was recruited to determine the effects of allele substitutions on the binding site of transcriptional regulators and splicing factors [56]. Using protein information, the SNAP server predicts the effect of nonsynonymous SNPs on protein function [57]. The miRWayDB database was utilized to experimentally validate miRNA pathway associations under pathophysiological conditions [58].

## 3. Results

### 3.1. Clinical and Demographic Characteristics of the Studied Subjects

Table 2 summarizes the clinical and demographic characteristics of BD patients and controls. No statistical differences were observed between the studied groups regarding age, gender, and BMI (*P* = 0.326, *P* = 0.899, and *P* = 0.745, respectively). The average age of BD onset was about 25.96 ± 9.71 years in our population. Approximately 183 (72.6%) patients were diagnosed with BDI, and the others were diagnosed with BDII (27.4%). There were no significant differences in age or gender between the BDI and BDII subgroups (*P* = 0.062 and 0.823, respectively). In addition, most patients were unemployed (59.1%) and had experienced mania (47.2%) at the time of diagnosis. About 34.1% of BD subjects presented with depression, and 18.7% simultaneously experienced mania and depression. Moreover, we found that 64.3% of BD patients had a family history of mood disorders in their first-degree relatives. We did not find any difference in the family history of mood disorders between the BDI and BDII subgroups (*p* = 0.689).

### 3.2. Genetic Association Analysis

Allelic and genotypic distribution of the studied SNPs is presented in Table 3. For all the studied SNPs, genotype distribution in the cases and controls was compatible with the Hardy-Weinberg equilibrium (HWE) (*P* value >0.05). The T allele of rs1261084C/T polymorphism significantly enhanced the risk of BD (OR = 1.36, 95% CI = 1.05 − 1.76, *P* = 0.021). The TT genotype in codominant 2 (TT vs. CC) models increased the risk of BD in our population (OR = 1.84, 95% CI = 1.12 − 3.02, *P* = 0.016, respectively). Similarly, the T allele in the dominant CC + CT vs. TT model enhanced BD risk by 1.61-fold (OR = 1.61, 95% CI = 1.06 − 2.45, *P* = 0.025). Regarding the rs10774053A/G polymorphism, the G allele (OR = 1.54, 95% CI = 1.19 − 1.99), as well as the GG genotype (OR = 1.57, 95% CI = 1.04 − 2.38, *P* = 0.032), enhanced the risk of BD in our population. Moreover, under the recessive (GG vs. AG + AA) and dominant (AA + AG vs. GG) modes of inheritance, increased BD risk was observed by 1.90 and 1.57–folds, respectively. For rs10466907G/T, the T allele was more frequent in BD subjects than in healthy subjects (OR = 1.33, 95% CI = 1.02 − 1.73, *P* = 0.034). In this case, the codominant 2 (TT vs. GG) model was correlated with enhanced risk of BD (OR = 1.94, 95% CI = 1.09 − 3.47, *P* = 0.025). Similarly, rs1625579A/C served as a risk factor for the onset of BD. The A allele of this SNP statistically increased the risk of BD by 1.47-fold (OR = 1.47, 95% CI = 1.14 − 1.91, *P* = 0.003). The CC genotype compared to AA genotype (codominant 2 model) caused a 2.12-fold increase in BD risk (OR = 2.12, 95% CI = 1.26 − 3.57, *P* = 0.004). Meanwhile, significant enhancement in BD risk was observed under the dominant AA + AC vs. CC (OR = 1.69, 95% CI = 1.08 − 2.63, *P* = 0.021) and recessive CC vs. AC + AA (OR = 1.64, 95% CI = 1.09 − 2.44, *P* = 0.016) contrasted genetic patterns.

Table 4 demonstrates the relationship between the genotype frequencies of studied variants and disease subtypes. Within-group comparison indicated a significant association between the frequency of GG genotype and GT genotypes of CACNA1C rs10466907G/T polymorphism among BDI and BDII cases (*P* value =0.014).

The interaction analysis of studied variants is shown in Table 5. In this regard, some interactions with frequencies under 1% (in either BD cases or healthy individuals) were excluded. Among all combined genotypes in the control group, the CT/AG/GT/AC genotype of rs1261084/rs10774053/rs10466907/rs1625579 polymorphisms was more frequent, hence considered the reference genotype. Both TT/AG/GT/AA and TT/GG/GT/AC combinations of genotypes strongly enhanced the risk of BD (OR = 5.24, 95% CI = 1.06 − 25.97, *P* = 0.036 and OR = 5.76, 95% CI = 1.17 − 25.25, *P* < 0.001, respectively).

### 3.3. Computational Findings

The genomic and transcriptomic sequences were obtained from the National Center for Biotechnology Information (NCBI), Ensembl, and UCSC Genome Browser databases for computational analyses. By employing the mirSNP database, we found that *TCF4* rs1261084C/T is likely to produce and disrupt some miRNA binding sites. Specifically, the T allele of this variation creates a de novo binding site for hsa-miR-105-3p, while the C allele can break the hsa-miR-356 binding site. In addition, both alleles of rs1261084C/T can enhance the affinity of TCF4 to hsa-miR-3151 and hsa-miR-3180 (Table 6). Regarding rs10466907G/T polymorphism, the T allele can create a new binding site for hsa-miR-561-3p, while the G allele does not affect the miRNA binding sites (Table 6). In addition, to explore the role of the miRNAs above, the miRWaDB was recruited. We found that hsa-miR-105 targets insulin receptor substrate protein1 (IRS1), the serine/threonine kinase Akt, and 3-Phosphoinositide-dependent protein kinase-1 (PDK1) genes are all contributing to the phosphatidylinositol 3-kinase (PI3K)/AKT signaling pathway (data not shown).

To determine the possible effects of rs10774053A/G polymorphism on splicing sites, the SpliceAid2 database was recruited. A 100 bp flanking region containing this SNP was introduced as a reference sequence. The results of this database revealed that rs10774053A/G developed a new splicing site in the presence of the G allele. In addition to the ETR-3 splicing factor shared between both A and G alleles, a SRp30c arginine/serine p splicing factor is created in the presence of the G allele (Figure 2).

ETR-3 contributes to the developmental regulation and stability of multiple miRNAs in the cytoplasm and nucleolus [43]. Furthermore, the SNAP2 database predicted the functional effects of sequence variants. We observed that methionine to valine substitution in position 1821 of CACNA1C protein potentially might alter the function of this protein (Figure 3).

A meaningful discrepancy in the free energy of A and/or C alleles of rs1625579 was noticed by the RNAfold database. A 20 bp flanking region was introduced as a template sequence up and downstream of the SNP position. In the presence of the A allele, miR-137 has been found to be more stable than the C allele. The amount of the free energy of the thermodynamic ensemble is -1.76 kcal/mol and -1.34 kcal/mol, regarding A and C alleles, respectively (Figure 4).

## 4. Discussion

In the current study, we found that most BD cases were of the BDI subtype. Moreover, a large proportion of BD patients were experiencing mania at the time of recruitment. Furthermore, 59.1% of the enrolled patients were unemployed, which might not be surprising. Bauer et al. reported that frequent symptoms of BD, especially depression, preclude full-time responsibilities outside the home and contribute to disability in these patients [59]. In another study, Owen and coworkers showed that the relationship between social interaction and bipolar-related experiences is complex; however, BD is responsible for damaging social relationships and is associated with loss of social control via extreme mood states [60]. Genotyping results revealed that rs1261084C/T, rs1077453A/G, rs1625579A/C, and rs10466907G/T variants conferred an increased BD risk in a sample of the Iranian population. The most powerful increase in the risk of BD was observed under the codominant model of rs10774053G/G (OR = 2.23). Overall, enhanced risk of BD was noticed under the codominant homozygous, dominant, and allelic models of TCF4 rs1261084C/T, codominant homozygous and allelic models of CACNA1C rs10466907G/T polymorphisms as well as codominant homozygous, dominant, recessive, and allelic models of the CACNA1C rs10774053A/G. Notably, the A allele of miR-137 rs1625579A/C significantly enhanced the risk of BD under the codominant homozygous, dominant, recessive, and allelic contrasted models. In addition, both TT/AG/GT/AA and TT/GG/GT/AC genotype combinations strongly increased the risk of BD in the participants.

Bioinformatics analyses indicated that the hsa-miR-105-3p binding site is created in the presence of the T allele, while the C allele disrupts a binding site related to hsa-miR-356. Moreover, the T allele of CACNA1C can create a new binding site for hsa-miR-561-3p. The rs10774053A/G polymorphism is likely to change the pattern of splicing sites in its position, while the G allele of this variant introduces a new splicing site for the SRp30c splicing factor. The M1821V substitution caused a functional change in the CACNA1C protein and must be validated using *in vitro* methods. We observed that the secondary structure of miR-137 is more stable in the presence of the A allele.

To the best of our knowledge, this is the first study to explore the association between SNPs in miR-137 and its downstream genes and BD risk. It is hypothesized that SNPs located in the 3′-untranslated region (3′-UTR) of genes, such as TCF4 rs1261084C/T and *CACNA1C* rs10466907G/T, can influence the miRNA binding sites and gene expression. Moreover, the CACNA1C rs10774053A/G is a missense variation and displays a change in amino acid (methionine to valine). Finally, rs1625579A/C is located in the pri-miR-137 region, where nucleotide exchange may affect the maturation process of miRNA. This might result in changes in miRNA expression and its regulatory pathways.

As a candidate gene, CACNA1C is located on chromosome 12p13.33 and encodes the Cav1.2 channel [61]. These types of channels enable the influx of extracellular Ca2+ upon depolarization. Cav1.2 channels are expressed in neuronal cells and play various pivotal functions, including regulating Ca2+ secretion [62]. The TCF4 encoding gene resides on chromosome 18q21.2 [63]. TCF4 is a transcription factor from the helix-loop-helix (HLH) family, regulating many different genes contributing to cell differentiation and neurodevelopment [64]. Some evidence revealed that mutations in the TCF4 gene were associated with Pitt-Hopkins syndrome, a rare mental disease known as mental retardation. In addition, deletions in this gene have been recognized as a risk factor for autistic-like behaviors [65, 66].

The miR-137 and its four putative target genes, including CACNA1C, TCF4, CSMD1, and C10orf26, have gained much attention as they are involved in a series of psychiatric conditions [67]. Additionally, luciferase-based reporter assay analysis confirmed these genes as experimentally validated targets of the miR-137 [37]. Differential expression studies showed that miR-137 was upregulated in patients suffering from SCZ compared to healthy controls [68]. New evidence suggests that the expression level of miR-137 and its downstream targets is strongly correlated with the development, differentiation, and maturation of the nervous system [69] and contributes to the etiology of BD [32]. In 2014, Duan et al. reported that a rare functional noncoding SNP at the GWAS-implicated miR-137/miR2682 locus might be associated with risk of SCZ as well as BD [70]. Using neuronal-like SH-SY5Y cells, Strazisar et al. discovered that miR-137 SNPs might impact synaptogenesis and neural transmission gene sets [71]. As an intronic variant of miR-137, rs1625579A/C is located on chromosome 1p21.3. It was previously shown that rs1625579A/C influences the risk of SCZ in a sample of the Chinese Han population [72]. An abnormal level of mature miR-137 was recently found in the cerebral cortex of patients carrying the T allele of miR-137 rs1625579A/C. However, the underlying mechanism by which this SNP dysregulates miR-137 processing is not clear yet [30].

In 2012, Whalley et al. showed that miR-137 rs1625579A/C SNP affects brain function in people at high genetic risk of BD [32]. In 2016, Zhang et al. performed a meta-analysis and found that this SNP enhances the risk of SCZ under allelic, recessive, and additive models [72]. Guan et al. showed that SNPs in miR-137 (rs1625579A/C) and its target gene, CACNA1C (rs10774053A/G and rs10466907G/T) polymorphisms, are associated with enhanced risk of SCZ risk in the Han Chinese population [17]. In agreement with these reports, we observed a positive association between CACNA1C SNPs and BD in our population. Moreover, we found a positive association between miR-137 rs1625579A/C SNP and BD risk. Another study by Lin et al. showed that CACNA1C rs10466907G/T affects cognitive recovery in patients with BD following a 6-week open-label trial [73].

As a novel schizophrenia risk variant at miR-137, the rs1625579A/C has been previously associated with SCZ; however, the results were inconclusive. In this connection, van Erp et al. reported that genotypes of the miR-137 rs1625579A/C variation are associated with dorsolateral prefrontal cortex hyperactivation, a condition that is considered a measure of brain inefficiency in SCZ cases [74]. By performing a meta-analysis on 2847 patients and 3018 controls of Chinese ancestry, Zhang et al. reported a significant association between this SNP and risk of SCZ under allelic T vs. G and recessive TT vs. GT + GG genetic patterns. In contrast, no significant link was observed between the SNP and SCZ under the dominant TT + GT vs. GG genetic model [72]. In 2013, Cummings et al. genotyped 821 cases with SCZ, schizoaffective disorder, and BDI. They proposed that risk allele carriers of the miR-137 rs1625579A/C had more cognitive deficits in terms of episodic memory and attentional control. In other words, mood-congruent psychotic symptoms and specific cognitive deficits were found to be significantly linked to this SNP [75]. In another study, Pu and Xiao pooled the genotypic results of 30843 Asian individuals and evidenced no statistical correlation between miR-137 rs1625579A/C and risk of SCZ [76].

In a study in 2016, Deniz Ozel et al. assessed genotype frequencies of the TCF4 gene rs9960767 polymorphism in 95 patients with BD and 108 healthy controls of a Turkish population. Their findings revealed that this variation does not appear to be an independent risk factor for BD; nonetheless, their findings could be biased due to the small size of the studied population [77]. Few reports have established the link between SCZ and TCF4 rs1261084C/T. Using multiplex polymerase chain reaction- (PCR-) SNPscan assay, Gao et al. genotyped 448 SCZ cases and 628 controls from a northwest Han Chinese population and found no significant link between TCF4 rs1261084C/T and the disease. However, by combining the results of their study with previously published reports, they found a noteworthy association between TCF4 rs1261084C/T and SCZ susceptibility [78]. Results of an investigation by Hui et al. indicated that another SNP in the TCF4 gene, rs2958182A/T, affected SCZ risk and was associated with lower cognitive performance in the language in these patients [79]. These observations suggest that this noncoding variation might contribute to the development of psychiatric diseases. Regarding the CACNA1C polymorphisms, only one report has highlighted the association of CACNA1C rs10466907 with BD. In their study, Lin et al. performed an open-label trial on 192 BD cases suffering a major depressive episode. They found that after 6 weeks, the rs10466907GT genotype did not significantly enhance the executive function total scores on the Wisconsin Card Sorting Test compared with carriers of the TT genotype [73]. These observations shed light on the contribution of CACNA1C SNPs to cognitive recovery from depression in patients diagnosed with BD. Another SNP in the CACNA1C encoding gene, rs10848683C/T, confers a higher risk of developing psychiatric disorders, including BD and SCZ, in subjects with family backgrounds [80]. Altogether, in our population, we observed significant links between the tested SNPs and BD risk. Hence, the miR-137 and its target genes might be involved in the pathogenesis of BD.

Our study has limitations. First, our sample size was modest, especially for stratified analyses. Hence, our findings should be validated through replicated studies using a larger sample size. Second, the frequency of the minor alleles of rs10774053 was not entirely consistent throughout the different populations in the world. This might be due to the limited sample size. According to our findings, the frequency of the minor alleles of rs1261084C/T, rs10774053A/G, rs10466907G/T, and rs1625579A/C were found to be 0.48, 0.45, 0.38, and 0.49. In addition, the frequency of genetic variations may be varied through different populations. For example, based on the information provided by the ensemble database (available at https://asia.ensembl.org/index.html), the T allele of rs1261084 is more frequent than the C allele in the majority of populations, even though it acted as the minor allele in our population. Moreover, in the case of rs10466907, the T allele is less frequent in the African and our populations; however, it cannot be applied to other populations. Finally, although stratified analyses were conducted, additional subtle stratified analyses should be done in further studies, e.g., in subgroups of early-onset and late-onset BD cases.

## 5. Conclusion

Our results provided evidence for the involvement of genetic variations in miR-137 and its target genes, TCF4 and CACNA1C, in the onset and development of BD. We have found that all the studied SNPs are positively associated with BD susceptibility. Future studies with a larger sample size are required to confirm these preliminary results. Further functional studies on determining the potential epistatic interactions between miR-137 and its putative targets would be desirable to elucidate the etiology of BD and discover novel strategies to treat this severe mental disorder.

## Figures and Tables

**Figure 1:** Gel electrophoretic separation of PCR products for (a) miR137 rs1625579, (b) CACNA1C rs10774053, (c) CACNA1C rs10466907, and (d) TCF4 rs1261084 polymorphisms.

**Figure 2:** The results of the SpliceAid2 server for predicting the effect of rs10774053A/G on the spicing sites. G allele introduced a new binding site for the SRp30c splicing factor. As shown, the rs10774053A/G SNP created a new splicing site in the presence of the G allele. In addition to the ETR-3 splicing factor shared between both alleles, the SRp30c arginine/serine p splicing factor is created in the presence of the G allele of this SNP. A positive score is assigned to a sequence that enhances exon definition, which can be either intronic splicing silencer (ISS) or exonic splicing enhancer (ESE) and localized to the above middle line. Accordingly, a negative score is assigned to a sequence that enhances intron definition, which can be either intronic splicing enhancer (ISE) or exonic splicing silencer (ESS), and is localized to the below-mentioned line.

**Figure 3:** Functional analysis of rs10774053A/G by SNAP server. The results showed that M1821V substitution might alter the function of CACNA1C.

**Figure 4:** The secondary structure of hsa-miR-137 regarding miR-137 rs1625579A/C. The results revealed that the local secondary structure of hsa-miR-137 is more stable in the presence of the A allele. The amount of the free energy of the thermodynamic ensemble is -1.76 kcal/mol and -1.34 kcal/mol, regarding A and C alleles, respectively. In the RNAfold server, each base is colored by the positional entropy and probability of forming pairs with paired bases and remaining unpaired bases. The red color represents the highest entropy and probability of forming pairs with paired bases, whereas, purple represents the lowest entropy.

**Table 1:** Designed primers for genotyping of the studied SNPs.

SNP	Genotyping method	Primer sequence	Annealing temperature (°C)	RE	Product size (bp)
rs1261084C/T	PCR-RFLP	F: CAAAGTAGATTGATGTCCATTCTAC	55	*FokI*	C: 405
		R: GCTCTGAACTGCACCAGTGTTTTCG			A: 204 + 201
rs10774053A/G	PCR-RFLP	F: GCACTCGGCTCTGAGAGGATGG	56	*MspI*	A: 402
		R: CCTGGGTCTTTGGCATTTGGC			C: 201 + 201
rs10466907G/T	ARMS-PCR	F (T-allele): TCTTATGTCAAAGCAATGAGACT	55	—	T or G: 250
		F (G-allele): TCTTATGTCAAAGCAATGAGACG			
		R (common): TACTTCCATCCAAGGGAGTCACT			
rs1625579A/C	Tetra-ARMS-PCR	FO: GTATGAGAACATCATGGGGTCAC	62	—	Outer band: 306
		RO: CCAAAGGTCTCTAGTGTGCTTGTAC			A or C: 192
		F (A-allele): GGAAGCTTATTAAACTGAGTTGGTT			
		F (C-allele): GGAAGCTTATTAAACTGAGTTGGTG			

F: forward; R: reverse; FO: forward outer; RO: reverse outer; SNP: single-nucleotide polymorphism; RFLP-PCR: restriction fragment length polymorphism polymerase chain reaction; ARMS-PCR: amplification refractory mutation system polymerase chain reaction; RE: restriction enzyme; BP: base pair.

**Table 2:** Clinical and demographic characteristics of BD patients and controls.

Parameter evaluated	BD (*n*, %) (mean ± SD)	BDI (*n*, %) (mean ± SD)	BDII (*n*, %) (mean ± SD)	Controls (*n*,%) (mean ± SD)	*P* value
Age (year)					
18-29	157 (62.3)	108 (59.0)	49 (71.0)	115 (54.0)	*P*_1_: 0.063
30-44	85 (33.7)	65 (35.5)	20 (29.0)	79 (37.1)	*P*_2_: 0.062
45-64	10 (4.0)	10 (5.5)	0	17 (8.0)	
>64	0	0	0	2 (0.9)	
Gender (female/male)	72/180	53/130	19/50	62/151	*P*_1_: 0.899 *P*_2_: 0.823
BMI (kg/m2)	23.25 ± 3.92	23.28 ± 4.23	23.19 ± 2.96	23.42 ± 2.80	*P*_1_: 0.745 *P*_2_: 0.547
Age at onset (year)	25.96 ± 9.71	25.84 ± 9.02	26.29 ± 11.40	—	*P*_2_: 0.050
Employment status					
Full-time worker	26 (10.3)	23 (12.6)	3 (4.3)	111 (81.0)	*P*_1_: <0.001
Part-time worker	36 (14.3)	28 (15.3)	8 (11.6)	51 (58.6)	*P*_2_: 0.109
Retired	8 (3.2)	4 (2.2)	4 (5.8)	0 (0)	
Unemployed	149 (59.1)	104 (56.8)	45 (65.2)	32 (17.7)	
Other	33 (13.1)	24 (13.1)	9 (13.0)	19 (38.8)	
Family history of mood disorder				—	*P*_2_: 0.689
Presence	162 (64.3)	119 (65.0)	43 (62.3)		
Absence	90 (35.7)	64 (35.0)	26 (37.7)		
History of suicide attempt				—	*P*_2_: 0.726
Presence	116 (46.0)	83 (45.4)	33 (47.8)		
Absence	136 (54.0)	100 (54.6)	36 (52.2)		
History of anxiety disorders				—	*P*_2_: 0.767
Presence	194 (77.0)	140 (76.5)	54 (78.3)		
Absence	58 (23.0)	43 (23.5)	15 (21.7)		
Hospitalization in past 12 months				—	*P*_2_: 0.712
Once	158 (62.7)	116 (63.4)	42 (60.9)		
Two or more	94 (37.3)	67 (36.6)	27 (39.1)		
Mood				—	*P*_2_: 0.880
Depressed	86 (34.1)	62 (33.9)	24 (34.8)		
Mania	119 (47.2)	88 (48.1)	31 (44.9)		
Mix	47 (18.7)	33 (18.0)	14 (20.3)		
Episodes of mania/hypomania (per year)				—	*P*_2_: 0.519
<4	191 (75.8)	142 (77.6)	49 (71.0)		
4-20	57 (22.6)	38 (20.8)	19 (27.5)		
>20	4 (1.6)	3 (1.6)	1 (1.4)		

BD: bipolar disorder; BMI: body mass index. *P* < 0.05 was considered statistically significant. P_1_: BD vs. control; P_2_: BDI vs. BDII.

**Table 3:** Allelic and genotypic distribution of miR-137 (rs1625579A/C), TCF4 (rs1261084C/T) and CACNA1C (rs10774053A/G, rs10466907G/T) polymorphisms.

SNP	BD, *n* (%)	Control, *n* (%)	Genetic model	OR (95% CI)	*P* value
rs1261084C/T					
CC	54 (21.4)	65 (30.5)		1 [reference]	
CT	114 (45.3)	93 (43.7)	Codominant 1	1.48 (0.94-2.32)	0.092
TT	84 (33.3)	55 (25.8)	Codominant 2	1.84 (1.12-3.02)	0.016
HWE (*P* value)	0.192	0.068	Dominant	1.61 (1.06-2.45)	0.025
			Recessive	1.44 (0.96-2.15)	0.078
Overdominant	1.07 (0.74-1.54)	0.733
C	222 (44.0)	217 (51.7)	Allelic	1 [reference]	—
T	282 (56.0)	203 (48.3)	Allelic	1.36 (1.05-1.76)	0.021
rs10774053A/G					
AA	56 (22.3)	66 (31.0)		1 [reference]	
AG	111 (44.0)	102 (47.9)	Codominant 1	1.28 (0.82-2.00)	0.274
GG	85 (33.7)	45 (21.1)	Codominant 2	2.23 (1.34-3.70)	0.002
HWE (*P* value)	0.089	0.632	Dominant	1.57 (1.04-2.38)	0.032
			Recessive	1.90 (1.25-2.89)	0.003
Overdominant	0.86 (0.59-1.24)	0.408
A	223 (44.2)	234 (54.9)	Allelic	1 [reference]	
G	281 (55.8)	192 (45.1)	Allelic	1.54 (1.19-1.99)	0.001
rs10466907G/T					
GG	69 (27.4)	74 (34.7)		1 [reference]	
GT	136 (54.0)	113 (53.1)	Codominant 1	1.29 (0.85-1.95)	0.224
TT	47 (18.6)	26 (12.2)	Codominant 2	1.94 (1.09-3.47)	0.025
HWE (*P* value)	0.164	0.085	Dominant	1.41 (0.95-2.10)	0.087
			Recessive	1.65 (0.98-2.77)	0.057
Overdominant	1.04 (0.72-1.50)	0.843
G	274 (54.4)	261 (61.3)	Allelic	1 [reference]	
T	230 (45.6)	165 (38.7)	Allelic	1.33 (1.02-1.73)	0.034
rs1625579A/C					
CC	44 (17.5)	56 (26.3)		1 [reference]	
AC	118 (46.8)	103 (48.4)	Codominant 1	1.46 (0.91-2.34)	0.119
AA	90 (35.7)	54 (25.3)	Codominant 2	2.12 (1.26-3.57)	0.004
HWE (*P* value)	0.620	0.631	Dominant	1.69 (1.08-2.63)	0.021
			Recessive	1.64 (1.09-2.44)	0.016
Overdominant	0.94 (0.65-1.35)	0.742
C	206 (40.9)	215 (50.5)	Allelic	1 [reference]	
A	298 (59.1)	211 (49.5)	Allelic	1.47 (1.14-1.91)	0.003

BD: bipolar disorder; SNP: single-nucleotide polymorphism; CI: confidence interval; OR: odd ratio; HWE: Hardy-Weinberg equilibrium. Codominant 1 and Codominant 2 represent the heterozygous and homozygous codominant models, respectively. *P* < 0.05 is considered statistically significant.

**Table 4:** Association of different genotype of the the studied variants with disease subtypes.

Disease type	Case genotypes of TCF4 rs1261084C/T			Test of sig	Within-group comparison	Case genotypes of CACNA1C rs10774053A/G			Test of sig	Within-group comparison
	CC *N* = 54	CT *N* = 114	TT *N* = 84			AA *N* = 56	AG *N* = 111	GG *N* = 85		
BDI	41 (22.4)	82 (44.8)	60 (32.8)	*X* ^2^: 0.384 *P*: 0.825	*P*_1_: 0.585 *P*_2_: 0.561 *P*_3_: 0.938	36 (19.7)	85 (46.4)	62 (33.9)	*X* ^2^: 2.83 *P*: 0.242	*P*_1_: 0.093 *P*_2_: 0.275 *P*_3_: 0.560
BDII	13 (18.8)	32 (46.4)	24 (34.8)			20 (29.0)	26 (37.7)	23 (33.3)		

Disease type	Case genotypes of *CACNA1C* rs10466907G/T			Test of sig	Within-group comparison	Case genotypes of miR-137 rs1625579A/C			Test of sig	Within-group comparison
	GG *N* = 69	GT *N* = 136	TT *N* = 47			AA *N* = 90	AC *N* = 118	CC *N* = 44		
BDI	57 (31.1)	90 (49.2)	36 (19.7)	*X* ^2^: 6.68 *P*: 0.036	*P*_1_: 0.014 *P*_2_: 0.425 *P*_3_: 0.184	65 (35.5)	82 (44.8)	36 (19.7)	*X* ^2^: 2.46 *P*: 0.292	*P*_1_: 0.668 *P*_2_: 0.226 *P*_3_: 0.117
BDII	12 (17.4)	46 (66.7)	11 (15.9)			25 (36.2)	36 (52.2)	8 (11.6)		

BD: bipolar disorder; BDI: bipolar disorder type I; BDII: bipolar disorder type II; P1: wild-type homozygote vs. heterozygote genotype; *P*_2_: wild-type homozygote vs. mutant homozygote; *P*_3_: heterozygote vs. mutant homozygote. *X*^2^ and *P* represent the amount of Chi-square and asymptotic significance (2-sided), respectively. *P* < 0.05 was considered statistically significant.

**Table 5:** Interaction analysis of the studied SNPs on BD risk.

rs1261084C/T	rs10774053A/G	rs10466907G/T	rs1625579A/C	BD (%)	Control (%)	OR (95% CI)	*P* value^∗^
CT	AG	GT	AC	7 (2.8)	11 (5.2)	1 [reference]	
CC	AA	GT	AA	7 (2.8)	2 (0.9)	5.50 (0.88-34.46)	0.03
CC	AA	GT	AC	2 (0.8)	7 (3.3)	0.45 (0.07-2.81)	0.36
CC	AG	GT	AC	5 (2.0)	8 (3.8)	0.98 (0.23-4.25)	0.72
CC	AG	GT	CC	3 (1.2)	8 (3.8)	0.59 (0.11-3.01)	0.52
CC	GG	GT	AC	8 (3.2)	3 (1.4)	4.19 (0.82-21.40)	0.08
CT	AA	GG	AC	4 (1.6)	5 (2.3)	1.26 (0.25-6.36)	0.76
CT	AA	GT	AC	6 (2.4)	4 (1.9)	2.36 (0.49-11.45)	0.28
CT	AG	GG	AC	7 (2.8)	5 (2.3)	2.20 (0.50-9.75)	0.28
CT	AG	GT	AA	11 (4.4)	8 (3.8)	2.16 (0.58-8.04)	0.24
CT	AG	GT	CC	9 (3.6)	6 (2.8)	2.36 (0.58-9.580	0.20
CT	GG	GG	AC	4 (1.6)	7 (3.3)	0.90 (0.19-4.24)	0.88
CT	GG	GT	AA	7 (2.8)	2 (0.9)	5.50 (0.88-34.46)	0.04
CT	GG	GT	AC	9 (3.6)	6 (2.8)	2.36 (0.58-9.58)	0.20
TT	AG	GG	AC	5 (2.0)	6 (2.8)	1.31 (0.29-5.98)	0.72
TT	AG	GT	AA	10 (4.0)	3 (1.4)	5.24 (1.06-25.97)	0.036
TT	AG	GT	AC	14 (5.6)	9 (4.2)	2.44 (0.69-8.66)	0.16
TT	AG	GT	CC	2 (0.8)	7 (3.3)	0.45 (0.07-2.81)	0.36
TT	GG	GT	AC	11 (4.5)	3 (1.4)	5.76 (1.17-25.25)	<0.001

OR: odd ratio; CI: confidence interval; BD: bipolar disorder. ^∗^*P* values were corrected for multiple testing. ^∗^*P* < 0.05 was considered statistically significant.

**Table 6:** The effect of 3′ UTR variants of TCF4 and CACNA1C on miRNA binding sites.

Gene	miRNA	SNP	Effect	Allele	Energy	Conservation
TCF4	Hsa-miR-105-3p	rs1261084	Create	C		
				T	-18.66	0.002
TCF4	Hsa-miR-356	rs1261084	Break	C	-22.47	0.002
				T		
TCF4	Hsa- miR-3151	rs1261084	Enhance	C	-23.24	0.036
				T	-22.26	0.036
TCF4	Hsa- miR-3180	rs1261084	Enhance	C	-19.77	0.028
				T	-21.15	0.028
CACNA1C	Hsa- miR-561-3p	rs10466907	Create	T	-6.39	0.040
				G		

SNP: single-nucleotide polymorphism; miRNA: microRNA.

## Data Availability

The raw data are available upon reasonable requests.
